The article "Effects of Laparoscopic versus Open Surgery for Advanced Gastric Cancer after Neoadjuvant Chemotherapy: A Meta-Analysis" was retracted in 2023. Reasons: signs of a paper mill; suspected computer-generated content; unreliable results or conclusions; concerns about the data.

# Effects of Laparoscopic versus Open Surgery for Advanced Gastric Cancer after Neoadjuvant Chemotherapy: A Meta-Analysis

**DOI:** 10.1155/2022/3255403

**Published:** 2022-06-18

**Authors:** Kun Huang, Jie Zhong, Dequan Jiang

**Affiliations:** ^1^Department of General Surgery, Central Hospital of Jiangjin District, Chongqing 400000, China; ^2^Department of General Surgery, Chongqing University Jiangjin Hospital, School of Medicine, Chongqing University, Chongqing 40000, China

## Abstract

**Objective:**

To evaluate the efficacy of laparoscopy and laparotomy after neoadjuvant chemotherapy in the treatment of advanced gastric cancer by meta-analysis.

**Methods:**

Cochrane Library, Embase, and PubMed were searched by computer until December 1, 2021. Literature was screened according to inclusion and exclusion criteria, and relevant data were extracted for meta-analysis using RevMan 5.3.

**Results:**

A total of 1027 patients from 11 literature studies were included in this study, including 413 patients in the laparoscopic group and 614 patients in the open group. Meta-analysis showed that the laparoscopic group had less intraoperative bleeding (SMD = −1.11; 95% CI: −1.75–0.47; *P*=0.0006), early postoperative exhaust (SMD = −0.45; 95% CI: −0.70–0.20; *P*=0.0004), and shorter postoperative hospital stay (SMD = 0.97; 95% CI: 1.69∼0.26; *P*=0.008), but had longer the operation time (SMD = 0.65; 95% CI: 0.52∼0.79; *P* < 0.00001). There was no significant difference in the number of lymph nodes dissected during operation (SMD = −0.45; 95% CI: −0.42–0.19; *P*=0.45), the incidence of surgical complications 30 days after operation (OR = 0.78; 95% CI: 0.53∼1.13; *P*=0.19), time of first defecation (MD = 0.00; 95% CI: −0.10∼0.10; *P*=0.98), and time of first postoperative feeding (MD = −0.05; 95% CI: −0.22∼0.12; *P*=0.54) between the two groups. For long-term prognosis, there was no significant difference in the 3-year overall survival rate after operation between the two groups (RR = 0.84; 95% CI: 0.63–1.12; *P*=0.23).

**Conclusion:**

Compared with the open stomach cancer surgery, laparoscopic gastric cancer surgery has less intraoperative blood loss, shorter hospitalization time, and advantages such as early rehabilitation, postoperative complications rate, and long-term survival, which confirmed the validity and security of the laparoscopic surgery.

## 1. Introduction

Gastric cancer is one of the most common malignant tumors in the world. In 2018, there were 1,034,000 new cases and 783,000 deaths of gastric cancer worldwide, accounting for the 5th and 3rd place, respectively, in the incidence and mortality of all cancers [1]. The proportion of early gastric cancer is relatively low, about 20%. Most of gastric cancers are already in the advanced stage when detected, and the overall 5-year survival rate is less than 50% [2]. Studies have shown that adjuvant chemotherapy (NAC) can reduce tumor size, increase R0 resection rate, and improve the prognosis of patients [3–5]. At present, surgery-based comprehensive treatment is the main mode of gastric cancer treatment [6], but open surgery causes great trauma, large amount of blood loss, and high incidence of complications, and some patients have poor tolerance to surgery and slow postoperative recovery [7–9]. In recent years, with the development of laparoscopic technology, laparoscopic gastric cancer surgery has become a research focus [10]. For advanced distal gastric cancer, NAC combined with laparoscopic radical gastrectomy does not increase complications, incidence and safety risks [9, 11].

The article "Effects of Laparoscopic versus Open Surgery for Advanced Gastric Cancer after Neoadjuvant Chemotherapy: A Meta-Analysis" was retracted in 2023. Reasons: signs of a paper mill; suspected computer-generated content; unreliable results or conclusions; concerns about the data.

In recent years, minimally invasive surgery for gastric cancer represented by laparoscopic radical gastrectomy has attracted wide attention. Kitano et al. [12] reported the world's first laparoscopic radical gastrectomy for gastric cancer in 1994 and gradually promoted it to the whole world thereafter. Laparoscopic radical gastrectomy for stage I distal gastric cancer was recommended by the 14th Edition of Japanese Gastric Cancer Guidelines [13]. With the rise of the technical level of the laparoscopic instruments' updates, laparoscopic D2 gastric cancer radical has gradually become the standard operation for treatment of cancer of the stomach [14]. A recent meta-analysis [15] also showed that preoperative neoadjuvant chemotherapy can improve the 5-year postoperative overall survival rate of gastric cancer patients and has no effect on the incidence of peroperative complications and mortality. However, the efficacy and safety of laparoscopic surgery for gastric cancer after neoadjuvant chemotherapy remain unclear. Li et al. [11] conducted a study to evaluate the short-term efficacy of laparoscopic or open distal gastrectomy in the treatment of advanced gastric cancer after neoadjuvant chemotherapy, and the results showed that the laparoscopic group had less surgical blood loss, low incidence of surgery-related complications, and significantly shortened postoperative hospital stay. The safety of laparoscopic surgery in patients with advanced gastric cancer undergoing NAC is an important issue faced by gastrointestinal surgeons.

There is still on debate that the efficacy of laparoscopic versus open surgery for advanced gastric cancer following neoadjuvant chemotherapy. To provide better evidence-based medical evidence, we conducted this meta-analysis to fully evaluate the short-term outcomes and long-term outcomes of laparoscopic versus open surgery for advanced gastric cancer following neoadjuvant chemotherapy.

The article "Effects of Laparoscopic versus Open Surgery for Advanced Gastric Cancer after Neoadjuvant Chemotherapy: A Meta-Analysis" was retracted in 2023. Reasons: signs of a paper mill; suspected computer-generated content; unreliable results or conclusions; concerns about the data.

## 2. Materials and Methods

### 2.1. Inclusion Criteria

Inclusion criteria were determined according to the PICOS principle (population, intervention, comparison, outcomes, and study design): (1) study population: advanced gastric cancer (cT_2-4a_N_0-3_M_0_ stage) was diagnosed by preoperative pathological gastroscopic biopsy and imaging results such as enhanced abdominal CT; (2) intervention measures: neoadjuvant chemotherapy and surgical treatment; (3) comparison type: laparoscopic surgery and open surgery; (4) outcome data: operative time, number of dissected lymph nodes, intraoperative blood loss, incidence of surgery-related complications 30 days after surgery, time of first postoperative exhaust, time of first postoperative defecation, time of first postoperative feeding, length of postoperative hospital stay, and overall survival at 3 and 5 years after surgery; (5) study design: case control study or clinical trial.

### 2.2. Exclusion Criteria

(1) Advanced patients with early or distant metastasis; (2) the full text is not available; (3) data of main indicators are incomplete.

### 2.3. Search Strategy

Two researchers searched PubMed, Cochrane Library, Embase, and other databases, respectively, and the time range was from the database establishment to December 1, 2021. Search terms included “gastric cancer,” “Laparoscopic Gastrectomy,” “Open Gastrectomy,” and “neoadjuvant Chemotherapy.”

### 2.4. Data Extraction and Literature Quality Evaluation

The obtained literature were imported into literature management software and screened according to inclusion and exclusion criteria. All data were obtained independently by two researchers from all eligible literature, and differences were resolved through discussion and negotiation. Data were extracted including author name, publication date, country and region, age, sample size, sex, and number of laparoscopic and open surgeries. The extracted outcome indicators included operative time, intraoperative blood loss, intraoperative lymph node dissection, postoperative complication rate 30 d, postoperative first exhaust time, postoperative first feeding time, postoperative length of hospital stay, and postoperative 3-year overall survival rate.

Randomized controlled trials (RCTS) were evaluated using the Cochrane Systematic Review Manual [16]. (1) Whether the allocation of hidden methods is reasonable; (2) blind method of subjects and intervention providers; (3) blind method of results evaluator; (4) the result data are incomplete; (5) report results selectively; (6) other biases. Each term was rated as low risk, unclear risk, or high bias risk. If each item is rated as low risk, the article is rated as low risk; if one or more items are rated as unknown risk, the article is rated as uncertain risk; and if one or more items are rated as high risk, the article is rated as high risk. Nonrandomized controlled trials (N-RCTs) were evaluated using the Newcastle–Ottawa scale, with a score ≥6 indicating high-quality studies [17].

The article "Effects of Laparoscopic versus Open Surgery for Advanced Gastric Cancer after Neoadjuvant Chemotherapy: A Meta-Analysis" was retracted in 2023. Reasons: signs of a paper mill; suspected computer-generated content; unreliable results or conclusions; concerns about the data.

### 2.5. Statistical Method

Statistical analysis was performed using RevMan 5.3. Rate ratios (RR) were used to evaluate category variables, and standardized mean difference (SMD) was used to evaluate continuous variables. Cochrane Q test and *I*^2^ statistics were used to evaluate the heterogeneity of the study. If *P* < 0.1 and/or I^2^ >50%, the heterogeneity was considered to be large, and the random effect model was applied for meta-analysis. If *P* > 0.1 and/or I^2^ <50%, the heterogeneity was considered small, and the fixed effect model was used for meta-analysis. When no standard deviation was reported in literature data, the standard deviation was estimated approximately according to the Hozo estimation method [18]. *P* < 0.05 was considered statistically significant.

## 3. Results

### 3.1. Literature Retrieval Results

A total of 715 articles were obtained through database retrieval, and 11 studies [11, 19–28] were obtained after exclusion according to exclusion criteria. There were 2 RCT studies [11, 20] and 9 N-RCT studies [19, 21–28], involving a total of 1027 patients, including 413 patients in the laparoscopic group and 614 patients in the open group. The literature screening process is shown in Figure 1, and the basic characteristics of the included literature are shown in Table 1.

### 3.2. Risk Assessment of Bias for Included Studies

Of the 2 included RCT studies, one [11] was low risk, and the other [20] was uncertain risk (Figure 2). The N-RCT scores of the 9 included studies [19, 21–28] were all ≥7, indicating that they were high-quality studies (Table 1).

### 3.3. Meta-Analysis

#### 3.3.1. Operation Time

The operation time was reported in 11 studies [11, 19–28], with no significant heterogeneity among studies (*P*=0.08; *I*^2^ = 41%). Fixed effect model analysis showed that the laparoscopic group had longer operation time (SMD = 0.65; 95% CI: 0.52–0.79; *P* < 0.00001), with statistical difference (Figure 3).

#### 3.3.2. Intraoperative Blood Loss

The intraoperative blood loss was reported in 11 studies [11, 19–28], with significant heterogeneity among studies (*P* < 0.000001; *I*^2^ = 95%). Random effect model analysis showed that the laparoscopic group had less intraoperative blood loss than that in the open group (SMD = −1.11; 95% CI:−1.75∼−0.47; *P*=0.0006), with statistical difference (Figure 4).

The article "Effects of Laparoscopic versus Open Surgery for Advanced Gastric Cancer after Neoadjuvant Chemotherapy: A Meta-Analysis" was retracted in 2023. Reasons: signs of a paper mill; suspected computer-generated content; unreliable results or conclusions; concerns about the data.

#### 3.3.3. The Number of Lymph Node Dissection

The number of lymph node dissection was reported in 11 studies [11, 19–28], with significant heterogeneity among studies (*P* < 0.000001; *I*^2^ = 80%). Random effect model analysis showed that there was no statistical difference between the laparoscopic group and open group in number of lymph node dissection (SMD = −0.45; 95% CI: −0.42∼0.19; *P*=0.45) (Figure 5).

#### 3.3.4. Complication Rate 30 Days after Operation

The complication rate 30 days after operation was reported in 11 studies [11, 19–28], with no significant heterogeneity among studies (*P*=0.24; *I*^2^ = 22%). Fixed effect model analysis showed that there was no statistical difference between the laparoscopic group and open group in complication rate 30 days after operation (RR = 0.84; 95% CI: −0.63–1.12; *P*=0.23). (Figure 6).

#### 3.3.5. The First Postoperative Exhaust Time

The first postoperative exhaust time was reported in 8 studies [11, 20, 21, 23–25, 27, 28], with significant heterogeneity among studies (*P*=0.02; *I*^2^ = 57%). Random effect model analysis showed that postoperative exhaust time of the laparoscopic group was earlier (SMD = −0.45; 95% CI: −0.70∼−0.20; *P*=0.0004), with statistical difference (Figure 7).

#### 3.3.6. The First Postoperative Feeding Time

The first postoperative feeding time was reported in 6 studies [11, 19, 21, 23, 27, 28], with no significant heterogeneity among studies (*P*=0.43; *I*^2^ = 0%). Fixed effect model analysis showed that the postoperative feeding time of the laparoscopic group was earlier (SMD = −0.45; 95% CI: −0.70∼−0.20; *P*=0.0004), with statistical difference (Figure 8).

#### 3.3.7. Postoperative Hospitalization Time

The postoperative hospitalization time was reported in 10 studies [11, 19–26, 28], with significant heterogeneity among studies (*P* < 0.00001; *I*^2^ = 96%). Random effect model analysis showed that postoperative hospitalization time of the laparoscopic group was shorter (SMD = −0.97; 95% CI: −1.69∼−0.26; *P*=0.008), with statistical difference (Figure 9).

#### 3.3.8. Three-Year Survival Rate

The three-year survival rate was reported in 3 studies [22, 26, 28], with significant heterogeneity among studies (*P*=0.007; *I*^2^ = 80%). Random effect model analysis showed that there was no statistical difference between the laparoscopic group and open group in three-year survival rate (RR = 1.04; 95% CI: −0.78∼1.39; *P*=0.78) (Figure 10).

### 3.4. Publication Bias Evaluations

Publication bias was evaluated by funnel plot, which showed that the studies on operative time and postoperative complications were basically symmetric, and the risk of publication bias was small (Figure 11).

The article "Effects of Laparoscopic versus Open Surgery for Advanced Gastric Cancer after Neoadjuvant Chemotherapy: A Meta-Analysis" was retracted in 2023. Reasons: signs of a paper mill; suspected computer-generated content; unreliable results or conclusions; concerns about the data.

### 3.5. Sensitivity Analysis

The heterogeneity of the five results was significant. Sensitivity analysis was conducted by eliminating each study in the index one by one. Among them, the data of intraoperative blood loss, intraoperative lymph node dissection, first postoperative exhaust time, and postoperative hospital stay were stable. In the meta-analysis of 3-year survival rate, heterogeneity (*I*^2^ = 0; *P*=0.71) decreased after the elimination of one study [26], and the fixed effect model was used for analysis, which had no significant impact on the results.

## 4. Discussion

Gastric cancer still is the malignant tumor that threatens human health seriously at present [29]. The 5-year survival rate of patients with stage I gastric cancer is 70%, while that of patients with stage IV gastric cancer is only 5% [30]. The treatment strategy of advanced gastric cancer is multidisciplinary treatment with surgery as the core. Adjuvant gastric infusion chemotherapy trial demonstrates for the first time that surgery combined with perioperative ECF chemotherapy (epirubicin + cisplatin + fluorouracil) significantly improves 5-year overall survival in patients with gastric cancer compared with surgery alone [31]. Recently, FLOT4 further improved the intensity of perioperative chemotherapy. FLOT (fluorouracil + oxaliplatin combined with docetaxel) being compared with ECF/ECX (epirubicin + cisplatin + fluorouracil infusion or oral capecitabine), the results showed that the overall survival rate and disease-free survival rate of the FLOT group were significantly improved. There was no significant difference in the rate of adverse reactions and mortality between the two groups [32]. With the development of relevant studies [33, 34], neoadjuvant chemotherapy for gastric cancer has been gradually promoted and recognized. In the US national comprehensive cancer network guidelines, neoadjuvant chemotherapy is recommended for advanced T2-4N0-3M0 gastric cancer [35]. Guideline of Chinese Society of Clinical Oncology for Gastric cancer recommends neoadjuvant chemotherapy for T3-4aN1-3M0 adenocarcinoma of gastroesophageal junction [36]. The advantages of preoperative neoadjuvant chemotherapy may include reducing the potential risk of tumor, reducing tumor size, increasing resectability, and eradicating occulent micrometastases [37]. However, the safety and efficacy of laparoscopic surgery in patients following neoadjuvant chemotherapy are unclear. Compared with open gastric cancer surgery, laparoscopic gastric cancer surgery has the advantages of small incision, light pain, short hospital stays, and early recovery [38]. The fibrotic response caused by chemotherapy and the loss of normal tissue plane caused by cytotoxicity present new technical challenges to laparoscopic surgery. Whether less trauma equates to better postoperative safety, chemotherapy completion, and survival benefits remains a key question in clinical practice. Whether laparoscopic surgery is better than open surgery has not been clearly determined. A total of 2 RCTS and 9 N-RCTs were included in this meta-analysis to evaluate the short-term effect and long-term prognosis of the two surgical methods for the treatment of advanced gastric cancer after neoadjuvant chemotherapy [39]. Results show that the laparoscopic surgery time is longer than open surgery, and this may be due to the fact that complex laparoscopic surgery operation has a long learning curve and is closely related to the performer experience, surgical skills. The results of a recently published study also showed that compared with inexperienced surgeons, the experienced surgeon line of laparoscopic radical gastrectomy operation time is shorter [39]. With the promotion of laparoscopic technology and the improvement of surgical proficiency, the time of laparoscopic surgery is expected to be shortened. The intraoperative blood loss in the laparoscopic group was less than that in the open group. Chemotherapy may lead to tissue fibrosis and damage to the anatomical plane, which may increase the risk of intraoperative complications. However, laparoscopic technology can provide a clear and enlarged field of vision during the operation, which is conducive to the operator to identify the anatomical levels and perform more delicate organ, vascular, and nerve operations [40]. There was no significant difference in the number of lymph node dissection between the two groups. Lymph node metastasis was an independent risk factor for tumor recurrence after radical gastrectomy. Higher number of lymph node dissection was more significant for advanced gastric cancer and accurate staging [41]. With the progress of endoscopic instruments such as fluorescence imaging laparoscopy and 3D laparoscopy, as well as the development and application of tracer materials such as carbon nanoparticles and indocyanine green, the efficiency of laparoscopic lymph node dissection is expected to be improved [42]. The first postoperative exhaust time and postoperative hospital stay in the laparoscopic group were shorter than those in the open group. Due to the fine operation and small trauma in the laparoscopic surgery, the intraoperative pull stimulation to the bowel can be reduced, which is conducive to the recovery of postoperative intestinal function. Besides, the incision is small, the postoperative pain is light, the early ambulation can be achieved, the recovery is fast, and the hospital stay is shortened [43]. The results of this study showed that there was no significant difference in the incidence of postoperative complications between the two groups, indicating the safety of laparoscopic surgery. In terms of long-term postoperative prognosis, the results of this study showed that there was no significant difference in the 3-year survival rate between the two groups, suggesting that the long-term efficacy of the two surgical procedures was similar.

The article "Effects of Laparoscopic versus Open Surgery for Advanced Gastric Cancer after Neoadjuvant Chemotherapy: A Meta-Analysis" was retracted in 2023. Reasons: signs of a paper mill; suspected computer-generated content; unreliable results or conclusions; concerns about the data.

This study has the following limitations: (1) among the included literature, 9 were retrospective studies and only 2 were randomized controlled studies, with publication bias; (2) preoperative neoadjuvant chemotherapy regiments are inconsistent in all studies, which may affect short-term prognosis and long-term survival of patients, and there may be significant heterogeneity among studies; (3) some included studies did not provide standard deviations, which were estimated approximately by the Hozo algorithm, and there may be outcome measurement bias; (4) the results of long-term prognosis of patients in the included studies are insufficient, and more reports of long-term follow-up results of studies are expected.

In conclusion, compared with the open stomach cancer surgery, laparoscopic gastric cancer surgery has less intraoperative blood loss, and shorter hospitalization time, and the advantages of the early rehabilitation, postoperative complications, and long-term prognosis confirmed the validity and security of laparoscopic surgery. However, it is worth noting that laparoscopic surgery is complicated, takes a long time, and has a long learning curve. Therefore, it is recommended that experienced surgeons perform neoadjuvant chemotherapy combined with laparoscopic surgery in the treatment of advanced gastric cancer. Meanwhile, more randomized controlled studies are expected to verify the results of this study in the future.

## Figures and Tables

**Figure 1:** Flowchart of the study selection.

**Figure 2:** Risk of bias summary for the included RCTs.

**Figure 3:** Forest plot comparing effect of operation time of laparoscopic operation and open operation for advanced gastric cancer.

**Figure 4:** Forest plot comparing the effect of intraoperative blood loss of laparoscopic operation and open operation for advanced gastric cancer.

**Figure 5:** Forest plot comparing effect of number of lymph node dissection of laparoscopic operation and open operation for advanced gastric cancer.

The article "Effects of Laparoscopic versus Open Surgery for Advanced Gastric Cancer after Neoadjuvant Chemotherapy: A Meta-Analysis" was retracted in 2023. Reasons: signs of a paper mill; suspected computer-generated content; unreliable results or conclusions; concerns about the data.

**Figure 6:** Forest plot comparing the effect of complication rate 30 days after operation of laparoscopic operation and open operation for advanced gastric cancer.

**Figure 7:** Forest plot comparing the effect of the first postoperative exhaust time of laparoscopic operation and open operation for advanced gastric cancer.

**Figure 8:** Forest plot comparing the effect of the first postoperative feeding time of laparoscopic operation and open operation for advanced gastric cancer.

**Figure 9:** Forest plot comparing the effect of the postoperative hospitalization time of laparoscopic operation and open operation for advanced gastric cancer.

**Figure 10:** Forest plot comparing the effect of the 3-year survival rate of laparoscopic operation and open operation for advanced gastric cancer.

**Figure 11:** Funnel plot of studies analyzing the effect of operative time and postoperative complications. (a) Operative time. (b) Postoperative complications.

**Table 1:** The baseline characteristics of the included studies.

Author,year	Country	Studytype	Operation	Sample	Gender(M/F)	Age (year)	Staging	Outcomes	Qualityassessment
Fujisaki, 2020	Japan	N-RCT	Laparoscopic surgery	20	13/7	71.5 ± 8.8	II-III	①②③④⑥⑦	8
			Open surgery	29	22/7	67 ± 8.5			

Hu, 2019	China	RCT	Laparoscopic surgery	23	10/13	61.4 ± 8.4	II-III	①②③④⑤⑦	Unclear risk
			Open surgery	27	14/13	64.1 ± 7.5			

Hu, 2022	China	N-RCT	Laparoscopic surgery	34	18/16	NA	II-III	①②③④⑤⑥⑦	8
			Open surgery	32	15/17	NA			

Khaled, 2021	Egypt	N-RCT	Laparoscopic surgery	41	20/21	62.29 ± 4.5	II-III	①②③④⑦⑧	8
			Open surgery	43	26/17	64 ± 10.7			

Li, 2016	China	N-RCT	Laparoscopic surgery	20	13/7	53.5 ± 9.2	I–III	①②③④⑤⑥⑦	8
			Open surgery	24	21/3	56 ± 9.2			

Li, 2019	China	RCT	Laparoscopic surgery	45	31/14	59 ± 3.25	I–III	①②③④⑤⑥⑦	Low risk
			Open surgery	50	35/15	61 ± 2			

Sheng, 2020	China	N-RCT	Laparoscopic surgery	45	23/22	62.12 ± 2.23	II-III	①②③④⑤⑦	7
			Open surgery	45	24/21	62.71 ± 2.16			

Wang, 2014	China	N-RCT	Laparoscopic surgery	68	39/26	52.9 ± 15.1	II-III	①②③④⑤⑦	7
			Open surgery	52	31/21	51.6 ± 8.2			

Wang, 2020	China	N-RCT	Laparoscopic surgery	49	34/15	54.4 ± 10.9	II-III	①②③④⑦⑧	8
			Open surgery	221	154/67	54.9 ± 11.3			

Wang, 2021	China	N-RCT	Laparoscopic surgery	23	18/5	60.09 ± 9.69	I–III	①②③④⑤⑥	8
			Open surgery	46	36/10	59.74 ± 8.65			

Xi, 2019	China	N-RCT	Laparoscopic surgery	45	36/9	57.1 ± 6.6	II-III	①②③④⑤⑦⑧	9
			Open surgery	45	33/12	59.6 ± 7.5			

## Data Availability

The simulation experiment data used to support the findings of this study are available from the corresponding author upon request.
